The article "A bibliometric analysis of global research on microbial immune microenvironment in melanoma from 2012 to 2022" was retracted in 2025. Reasons: unreliable results or conclusions; concerns about the data.

# A bibliometric analysis of global research on microbial immune microenvironment in melanoma from 2012 to 2022

**DOI:** 10.1111/srt.70017

**Published:** 2024-08-21

**Authors:** Lin Sun, Jianghui Ying, Rong Guo, Lingling Jia, Hongyi Zhang

**Affiliations:** ^1^ Department of Radiotherapy Yantaishan Hospital Shandong China; ^2^ Department of Plastic Surgery Shanghai East Hospital, Tongji University School of Medicine Shanghai China

**Keywords:** immune microenvironment, melanoma, microbes, microbial microenvironment, tumor immunotherapy

## Abstract

**Background:**

Melanoma is an aggressive malignancy primarily impacting the skin, mucous membranes, and pigment epithelium. The tumor microbial microenvironment encompasses both the microorganisms inhabiting the tumor vicinity and the environmental factors influencing their interactions. Emerging evidence highlights the pivotal role of the microbial immune microenvironment in melanoma.

**Methods:**

We conducted an extensive review of scholarly works published from 2012 to 2022, utilizing The Web of Science Core Collection. Subsequently, we employed analytical tools such as VOSviewer, CiteSpace, and the R programming language to scrutinize prevailing research patterns within this domain.

**Results:**

A sum of 513 articles were pinpointed, with notable input coming from the United States and China. Harvard University stood out as the top‐contributing institution, while the journal Science received the most citations. Current research within this sphere chiefly focuses on two principal domains: the gut microbiota and the PD‐L1 pathway concerning melanoma treatment.

**Conclusion:**

The study offers an extensive analysis and overview of the worldwide research landscape concerning the immune microenvironment with a focus on microbes in melanoma. It underscores the promising prospects for harnessing the microbial immune microenvironment's potential in melanoma. These findings furnish valuable insights and guidance for advancing scientific inquiry and refining clinical approaches within this dynamic field.

## 1 INTRODUCTION

Melanoma, an exceedingly malignant tumor, arises from the degeneration of melanocytes, a majority of which stem from typical moles and pigmented patches, and frequently manifest in skin tissues. ^1^ Compared with other common malignant tumors,^2^ melanoma has a lower incidence, but it is one of the fastest‐growing malignant tumors.^3^ Melanoma has the potential for both lymphatic and hematogenous metastasis during its early stages, leading to a dismal prognosis with a 5‐year survival rate of merely 10%. Standard therapeutic approaches encompass surgical intervention, radiation therapy, chemotherapy, and biological immunotherapy. Surgical resection is highly effective, curing approximately 90% of melanomas in their initial stages. However, as melanomas advance, the efficacy of treatments is typically suboptimal.^4^

The article "A bibliometric analysis of global research on microbial immune microenvironment in melanoma from 2012 to 2022" was retracted in 2025. Reasons: unreliable results or conclusions; concerns about the data.

The immune microenvironment, often referred to as the tumor immune microenvironment, encompasses the neighboring milieu of tumor cells, comprising microorganisms, adjacent blood vessels, immune cells, a spectrum of signaling molecules, and the extracellular matrix.^5^ The tumor maintains a close and dynamic relationship with this milieu, continuously engaging with it. By releasing cellular signaling molecules, promoting tumor angiogenesis, and inducing immune tolerance, the tumor can significantly influence its microenvironment. Concurrently, immune cells within the microenvironment can exert influence on the growth and progression of cancer cells. Notably, tumor tissues harbor various microorganisms, such as bacteria, fungi, viruses, and chlamydia. These constituents profoundly impact the initiation, advancement, metastasis, and immune responses related to tumors. This microorganism‐driven immune microenvironment is also recognized as the “tumor microbiome.”^6^

A growing body of evidence underscores the tight correlation between the immune microenvironment influenced by microbes (termed the tumor microbiome microenvironment) and the onset and progression of melanoma. Notably, the composition of the tumor microbiome varies across patients with differing survival rates, holding promise as a potential prognostic indicator.^7^ In a study by Alexandra Snyder and team,^8^ an analysis of tumor antigen epitopes in melanoma patients with distinct prognoses revealed homology between certain tumor neoantigen epitopes and microbial epitopes. Intriguingly, a positive association was observed between higher homology and improved clinical prognosis. This observation implies the presence of antigen mimicry within tumors, potentially impacting immune responses. In addition, they found that beneficial bacteria in the gut microbiome, such as probiotics, can participate in the treatment of metastatic melanoma by regulating immune checkpoint inhibitors (ICIs) and MAPK pathways.

Bibliometrics is a quantitative analysis of the internal connections and distribution patterns among published literature based on parameters such as country, institution, and author, using mathematical and statistical methods.^9^, ^10^ The objective is to investigate the present research status, focal points, and upcoming directions within a specific domain. Over the past few years, scholarly interest in understanding the impact of the microbe‐related immune microenvironment in melanoma has escalated significantly, paralleled by a sharp rise in the volume of pertinent literature. However, bibliometric studies in this field have not been reported yet. Within this investigation, we conducted a comprehensive search and analysis of scholarly reports regarding the influence of the microbe‐related immune microenvironment in melanoma, utilizing the Web of Science (WoS) database spanning from 2012 to 2022. We performed statistical analyses on the publications, institutions, and keywords, enabling the visualization of prevailing trends within this domain. This analysis offers valuable insights to guide forthcoming research endeavors.

The article "A bibliometric analysis of global research on microbial immune microenvironment in melanoma from 2012 to 2022" was retracted in 2025. Reasons: unreliable results or conclusions; concerns about the data.

## 2 MATERIALS AND METHODS

### 2.1 Data collection

We amassed pertinent literature concerning the influence of microbial‐related immune microenvironments in melanoma within the timeframe of 2012 to 2022, utilizing The Web of Science Core Collection (WoSCC). The search strategies were precisely defined as follows: TS = (Melanoma* OR Malignant Melanoma*) AND TS = (Microbiota* OR Microbes OR Microbial Communit* OR Microbial Community Composition* OR Microbial Community Structure* OR Microbiome* OR Human Microbiome* OR Microorganism* OR Microbiology OR Microbial) AND TS = (Immun* microenvironment OR Microenvironment of immun*) AND Publication Date = (2011‐01‐01 to 2021‐12‐31) AND Language = (English). Following this, manual screening of studies concerning the microbiome, immune microenvironment, and melanoma was conducted. For a comprehensive overview of the search process and specifics regarding the included studies, refer to Figure 1. The eligible article types included reviews and original articles. The data were independently retrieved and analyzed by both the primary and secondary authors. This encompassed gathering information such as the number of publications and citations, titles, countries/regions, affiliations, and related details from WoSCC for subsequent in‐depth analysis.

**FIGURE 1:** The screening process of the literature.

### 2.2 Bibliometric analysis

Bibliometric analysis employed various tools, including Microsoft Excel 2022, VOSviewer (version 1.6.17), CiteSpace V (version 6.2.2), and the R language package. The analysis was facilitated using the online tool available at http://www.bioinformatics.com.cn/srplot. Microsoft Excel 2022 was utilized for generating publication and citation yearbooks, utilizing data sourced from WoSCC. VOSviewer visualized bibliometric networks or density maps of collaborations among countries and organizations, journal links, and keyword co‐occurrence. CiteSpace V employed cooperation and clustering analysis among authors, as well as a large number of reference and keyword data. Utilizing the R language package, we generated the geographical distribution of worldwide publications, identified the top 10 productive institutions, and constructed a radar chart illustrating journals' contributions. Additionally, the most recent Impact Factor (IF) was sourced from the latest iteration of the Journal Citation Reports (JCR, 2022).

The article "A bibliometric analysis of global research on microbial immune microenvironment in melanoma from 2012 to 2022" was retracted in 2025. Reasons: unreliable results or conclusions; concerns about the data.

## 3 RESULTS

### 3.1 Global contributions and overall distributions

We identified a sum of 513 original articles and reviews associated with the microbial immune microenvironment in melanoma. The counts for publications and citations have consistently trended upward since 2012 (publications = 4, citations = 11), with minor downturns noted in 2014 and 2022. Notably, 2021 saw a pinnacle in publications (publications = 44), while 2022 marked the zenith in citation numbers (Figure 2A). The swift escalation in both publications and citations underscores the escalating attention researchers globally are dedicating to this domain.

**FIGURE 2:** (A) The number of publications and citations over the past decade; (B) A global map illustrating publication quantities by country; (C) The citation count in the top five countries each year; (D) The publication count in the top five countries annually.

Based on the country/region distribution map of publications (Figure 2B) and the leading 10 countries/regions contributing the most publications (Table 1), the foremost three countries include the United States (*n* = 80, 43.96%), China (Mainland China, subsequently referred to as China) (*n* = 62, 34.07%), and Germany (*n* = 13, 7.14%). Throughout the period from 2012 to 2022, both China and the United States exhibited a consistent upward trajectory in annual publications and citations, significantly outpacing other nations. Interestingly, although China and the United States are neck and neck in terms of publication numbers, with China even surpassing the United States in 2021, the citation rate for articles from the United States is significantly higher than that of China. Moreover, in the preceding decade, the aggregate publications (*n* = 142) and citations (*n* = 14 294) stemming from China and the United States have notably exceeded the cumulative from the remaining three countries (*n* = 30, *n* = 1764) (Figure 2C, D). Notably, the network map illustrating collaborative efforts between countries (Figure 3A) underscores the strong collaboration and central positioning of China and the United States within the multi‐country collaboration network. In summary, both China and the United States distinctly lead in this field, evident by their substantially higher publication and citation numbers concerning the microbial immune microenvironment in melanoma compared to other nations. Additionally, they serve as central nodes for collaborative efforts among multiple countries.

The article "A bibliometric analysis of global research on microbial immune microenvironment in melanoma from 2012 to 2022" was retracted in 2025. Reasons: unreliable results or conclusions; concerns about the data.

**TABLE 1:** Contributed publications in the top 10 countries.

Country	Publications	Citations	Average citation rate	% of	H‐index
USA	80	10 595	132.4	43.96	34
CHINA	62	3830	61.7	34.07	24
GERMANY	13	1118	86	7.14	10
ITALY	9	497	55.2	4.95	8
ENGLAND	8	237	29.6	4.40	7
FRANCE	8	2677	334.6	4.40	6
FINLAND	6	216	36	3.30	6
CANADA	5	143	28.6	2.75	3
ISRAEL	5	302	60.4	2.75	4
SWEDEN	5	3275	655	2.75	4

**FIGURE 3:** (A) The collaboration network among countries; (B) A radar chart showcasing the publication and citation counts per institution; (C) The collaboration network among institutions; (D) The collaboration heatmap among institutions.

### 3.2 Institutional and author analysis

In scrutinizing publication institutions, a comprehensive total of 1132 institutions engaged in scientific research concerning the microbial immune microenvironment in melanoma. The top 10 institutions, based on publication output, are detailed in Table 2. Harvard University leads with the highest productivity (*n* = 12), followed by the University of California System (*n* = 10) and the University of Texas System (*n* = 10). As for citations, Institut National De La Sante Et De La Recherche Medicale Inserm (*n* = 2820), University Of Texas System (*n* = 2519), and Harvard University (*n* = 1959) rank as the most cited institutions (Figure 3B). Subsequently, we utilized VOSviewer to conduct an in‐depth analysis and visualization of the extended network and density map illustrating institutional collaboration (Figure 3C, D). Notably, Harvard Medical School, The University of Texas MD Anderson Cancer Center, Sichuan University, and the University of Helsinki emerge as the most prominent research centers with the closest interconnections to other institutions.

**TABLE 2:** Top 10 institutions with the most publications.

Institutions	Country	Publications	Citations	Average citation rate	H‐index
Harvard University	USA	12	1959	163.2	11
University of California System	USA	10	578	57.8	8
University of Texas System	USA	10	2519	251.9	7
Harvard Medical School	USA	9	1820	202.2	9
National Institutes of Health Nih USA	USA	7	764	109.1	6
Utmd Anderson Cancer Center	USA	7	987	141	6
Chinese Academy of Sciences	CHINA	6	291	48.5	5
Institut National DE LA Sante ET DE LA Recherche Medicale Inserm	FRANCE	6	2820	470	6
North Carolina State University	USA	6	694	115.7	6
Sichuan University	CHINA	6	85	14.2	5

#### 3.2.1 Author analysis

In an examination of authors contributing to publications on the microbial immune microenvironment in melanoma, a collective total of 1640 authors have made substantial contributions. Table 3 delineates the top 10 authors based on their publication output. Zhuhao Gu is the foremost productive author, boasting five published papers in this field. In terms of citation count, Wargo Jennifer A holds the most influence, garnering a remarkable total of 943 citations. Analyzing the expansive collaboration network among authors, central positions are occupied by Zhen Gu, Xuesi Chen, and Steinmetz, Nicole F, signifying that the volume of publications, to a certain degree, reflects the level of collaboration among authors (Figure 4A).

The article "A bibliometric analysis of global research on microbial immune microenvironment in melanoma from 2012 to 2022" was retracted in 2025. Reasons: unreliable results or conclusions; concerns about the data.

**TABLE 3:** Top 10 authors with the most publications.

Author	Country	Documents	Citations	Average citation rate	H‐index
Gu, Zhuhao	CHINA	5	636	127.2	5
Chen, Xuesi	CHINA	4	242	60.5	3
Hemminki, Akseli	FINLAND	4	149	37.3	4
Hu, Quanyin	CHINA	4	565	141.3	4
Steinmetz, Nicole F.	USA	4	90	22.5	4
Wang, Chao	CHINA	4	436	109	4
Wang, Jinqiang	CHINA	4	563	140.8	4
Wang, Yi	CHINA	4	215	53.8	4
Wargo, Jennifer A	USA	4	943	235.8	4
Bridle, Byram W	CANADA	3	9	3	1

**FIGURE 4:** (A) Extensive collaboration network among authors. (B) Radar graph of publications and citations by journal.(C)The collaboration network graph of various journals.(D)The collaboration network heat map of various journals.

### 3.3 Journal analysis

A comprehensive total of 115 journals have accepted and published articles about the microbial immune microenvironment in melanoma. Table 4 provides an overview of the top 10 journals based on their publication output. ADVANCED MATERIALS (IF = 32.09), CANCERS (IF = 6.58), and NATURE COMMUNICATIONS (IF = 17.7) are the highest publishing journals, each with five articles published. SCIENCE, with an impact factor of 83.8, is the highest impact journal among all journals. SCIENCE (*n* = 5009) is the most cited journal, followed by ADVANCED MATERIALS (*n* = 536) and FRONTIERS IN IMMUNOLOGY (*n* = 228) (Figure 4B). (SCIENCE not only has the highest impact factor but also the highest citation count.) All journals belong to JCR Q1. Then, a network graph and density plot of journal collaboration were analyzed (Figure 4C, D). As shown in the figure, ADVANCED MATERIALS, FRONTIERS IN IMMUNOLOGY, JOURNAL OF IMMUNOLOGY, and CANCERS have the closest connections with other journals, and they are the publishing centers in this field of research. Therefore, the publishing volume and citation count of journals can to some extent determine the degree of collaboration between journals.

**TABLE 4:** Top 10 journals with the most publications.

Journal	Documents	Citations	Average citation rate	IF (2021)	JCR Partition
Advanced Materials	5	536	107.2	32.09	Q1
Cancers	5	73	14.6	6.58	Q1
Nature Communications	5	154	30.8	17.7	Q1
Biomaterials	4	186	46.5	15.3	Q1
Frontiers in Immunology	4	228	57	8.8	Q1
Immunotherapy	4	119	29.8	4	Q1
Journal of Immunology	4	82	20.5	5.4	Q1
Nano Today	4	36	9	19	Q1
Science	4	5009	1252.2	83.8	Q1
ACS Applied Materials Interfaces	3	20	6.67	10.4	Q1

The article "A bibliometric analysis of global research on microbial immune microenvironment in melanoma from 2012 to 2022" was retracted in 2025. Reasons: unreliable results or conclusions; concerns about the data.

### 3.4 Cited and co‐cited references analysis

Analyzing citations and co‐citations in the literature offers insights into the most influential research within the field, thus guiding the fundamental direction of future research. Table 5 showcases the top 10 most cited publications, while Table 6 presents the top 10 co‐cited publications. The article by Bertrand Routy et al. holds the highest citation count (*n* = 2716), while V Gopalakrishnan et al.’s work is the most co‐cited (*n* = 25). Notably, frequent mutual citations were observed among other publications (Figure 5A). In their study, Gopalakrishnan et al.^11^ investigated the microbial composition of the oral and gut microbiome in melanoma patients undergoing anti‐PDL‐1 (anti‐programmed cell death 1 protein) immunotherapy. They conducted an immunological analysis of the patients' fecal microbiota and observed that individuals with a healthy gut microbiome exhibited improved anti‐tumor immune function. However, resistance to anti‐PDL‐1 therapy remains a common challenge in melanoma treatment. Davar et al. conducted a clinical trial involving 15 melanoma patients, implementing fecal microbiota transplantation (FMT) to modulate the gut microbiome and overcome resistance to anti‐PDL‐1 therapy. This intervention effectively regulated the microbiome‐induced resistance mechanism within the immune microenvironment of melanoma.^12^

**TABLE 5:** Top 10 publications with the most citations.

Title	Journal	IF	Publication year	Total citations
Gut Microbiome Influences Efficacy Of PD‐1‐Based Immunotherapy Against Epithelial Tumors	Science	63.83	2018	2716
Commensal Bifidobacterium Promotes Antitumor Immunity And Facilitates Anti‐PD‐L1 Efficacy	Science	63.83	2015	2234
Signatures Of T Cell Dysfunction And Exclusion Predict Cancer Immunotherapy Response	Nature Medicine	87.24	2018	1555
Tertiary Lymphoid Structures Improve Immunotherapy And Survival In Melanoma	Nature	69.50	2020	751
Combination Delivery Of TGF‐Beta Inhibitor And IL‐2 By Nanoscale Liposomal Polymeric Gels Enhances Tumour Immunotherapy	Nature Materials	47.66	2012	299
Fecal Microbiota Transplant Overcomes Resistance To Anti‐PD‐1 Therapy In Melanoma Patients	Science	63.83	2021	386
PD‐1 And PD‐L1 Antibodies In Cancer: Current Status And Future Directions	Cancer Immunology Immunotherapy	6.63	2017	217
Injectable Bioresponsive Gel Depot For Enhanced Immune Checkpoint Blockade	Advanced Materials	32.09	2018	210
Gut Microbiota Promotes Tumor Growth In Mice By Modulating Immune Response	Gastroenterology	33.88	2018	198
PD‐1 Blockade Cellular Vesicles For Cancer Immunotherapy	Advanced Materials	32.09	2018	164

The article "A bibliometric analysis of global research on microbial immune microenvironment in melanoma from 2012 to 2022" was retracted in 2025. Reasons: unreliable results or conclusions; concerns about the data.

**TABLE 6:** Top 10 publications with the most co‐citations.

Title	Journal	IF	Publication year	Co‐citations number
Gut microbiome modulates response to anti‐PD‐1 immunotherapy in melanoma patients	Science	63.83	2018	25
The commensal microbiome is associated with anti‐PD‐1 efficacy in metastatic melanoma patients	Science	63.83	2018	20
Gut microbiome influences efficacy of PD‐1‐based immunotherapy against epithelial tumors	Science	63.83	2018	19
Oncolytic Virotherapy Promotes Intratumoral T Cell Infiltration and Improves Anti‐PD‐1 Immunotherapy	Cell	66.85	2017	17
Commensal Bifidobacterium promotes antitumor immunity and facilitates anti‐PD‐L1 efficacy	Science	63.83	2015	16
Cancer immunotherapy using checkpoint blockade	Science	63.83	2018	15
Anticancer immunotherapy by CTLA‐4 blockade relies on the gut microbiota	Science	63.83	2015	15
Pembrolizumab versus Ipilimumab in Advanced Melanoma	The New England journal of medicine	176.08	2015	12
Melanoma‐intrinsic β‐catenin signalling prevents anti‐tumour immunity	Nature	69.50	2015	12

**FIGURE 5:** (A) A network diagram displaying highly cited and co‐cited articles; (B) The top nine references with the most prominent citation bursts; (C) Cluster analysis of keyword co‐citations; (D) Timeline clustering of keywords.

Utilizing the co‐citation network, a reference burst analysis was conducted, presenting the top nine co‐cited references with the most pronounced citation bursts, as illustrated in Figure 5B. One of the prominent articles revealed in the burst analysis was authored by Ayelet and the team. Their study involved anti‐tumor experiments on melanoma‐afflicted mice, demonstrating that oral administration of bifidobacterium effectively enhances the anti‐tumor function of CD8+ T cells. This approach achieves immune regulation of tumors by modulating the tumor immune microenvironment.^13^ Subsequently, title clustering analysis was executed to succinctly summarize the referenced articles within the co‐citation network, aiming to comprehend the forefronts of this domain. The analysis led to the identification of fourteen distinct clusters from the co‐citation network, encompassing topics such as gut microbiota, rational combination, advanced melanoma resistance mechanisms, pdl‐1 pathway, intestinal microbiota regulation, commensal bifidobacterium, bacteria‐based cancer therapy, and cancer cell, among others (Figure 5C). Analyzing the timeline clustering (Figure 5D), it is evident that recent research has predominantly focused on gut microbiota, advanced melanoma resistance mechanisms, regulatory antitumor strategies, and bacteria‐based cancer therapy.

The article "A bibliometric analysis of global research on microbial immune microenvironment in melanoma from 2012 to 2022" was retracted in 2025. Reasons: unreliable results or conclusions; concerns about the data.

### 3.5 Analysis of keywords

The co‐occurrence analysis of keywords elucidates the inherent interconnections between terms within the microbial immune microenvironment in the melanoma domain. Employing VOSviewer, we visually represented the expansive network of co‐occurring keywords (Figure 6A). Notably, immunotherapy, cancer, and PDL‐1 blockade demonstrated the most robust correlations with other keywords, positioned centrally in the mutually cited keywords network. Concurrently, melanoma, cancer immunotherapy, and microbiome emerged as the author's keywords with the most pronounced correlations (Figure 6B).

**FIGURE 6:** (A) An extensive network reflecting co‐occurrence of keywords; (B) The author's keywords demonstrating the strongest correlation; (C) The keyword clustering network analysis; (D) Timeline clustering of reference keywords.

Delving into the analysis of keyword clustering network, we identified eight distinct clusters within the co‐occurrence keyword network, encompassing areas like microenvironment, gut microbiota, cancer immunotherapy, anticancer therapy, drug resistance, drug delivery, and growth (Figure 6C). Additionally, investigating the timeline clustering of reference keywords (Figure 6D), it is evident that gut microbiome, metastatic melanoma, and cancer immunotherapy have remained the primary research focus of scholars since 2012.

## 4 DISCUSSION

Melanoma, a perilous form of skin cancer, manifests as a malignant tumor within the skin. ^14^ Melanoma originates from melanocytes in the skin, which are responsible for producing pigment and helping to protect the skin from damage caused by sunlight. However, if these cells become abnormal, they may start to grow uncontrollably and form a tumor. The exact cause of melanoma is still not fully understood, but sunlight and ultraviolet radiation are among its main risk factors. Other risk factors include drug exposure, family history, and congenital lesions.^15^ The diagnosis of melanoma usually requires histological examination. Upon melanoma diagnosis, it is essential to undergo magnetic resonance imaging (MRI) and computed tomography (CT) scans to ascertain potential metastasis of the tumor to other body regions. The treatment of melanoma depends on the severity of the tumor and the extent of its spread and typically includes surgical removal, radiation therapy, and chemotherapy.^16^ Although melanoma is a very dangerous tumor, early diagnosis and treatment can greatly improve survival rates. Consequently, routine skin examinations play a vital role in the timely identification and management of melanoma.

The article "A bibliometric analysis of global research on microbial immune microenvironment in melanoma from 2012 to 2022" was retracted in 2025. Reasons: unreliable results or conclusions; concerns about the data.

The immune microenvironment refers to a complex microenvironment surrounding the tumor, composed of immune cells, cytokines, chemokines, blood vessels, and extracellular matrix.^17^ The term denotes the reciprocal interplay between tumor cells and the organism's immune system. The microbial immune microenvironment is the result of interactions between microbes and the immune system within an organism, encompassing microbial communities, immune cells, and diverse components across body regions such as the gut, skin, and oral cavity. This intricate microenvironment significantly influences immune system development and function. There are numerous microbial communities in the human body, and their interaction with the immune system can regulate immune system balance and function. As an illustration, specific microorganisms can modulate immune responses and balance immune tolerance by regulating T‐cell differentiation and function.^18^ Concurrently, the immune system plays a crucial role in preserving overall body health by recognizing and eliminating atypical microbial entities. In recent years, research on the microbial immune microenvironment has become one of the hotspots in the field of immunology. Through a deeper understanding of the microbial immune microenvironment, researchers can better understand the function and regulation mechanism of the immune system, introducing novel concepts and methodologies for disease treatment and prevention.

The microbial immune microenvironment profoundly influences the onset and progression of melanoma. Research suggests that an imbalance in gut microbiota might disrupt the immune microenvironment of melanoma, rendering it more susceptible to immune evasion.^19^ Additionally, specific microorganisms can impact the advancement and prognosis of melanoma by modulating immune system responses.^20^ For example, certain probiotics can augment the immune response by regulating T cell differentiation and function, thereby decelerating melanoma progression.^21^ In summary, the microbial immune microenvironment significantly contributes to melanoma onset and development, yet a comprehensive understanding of the precise mechanisms necessitates further investigation. Bibliometric analysis has very strong advantages in this area and is widely used in the study of many skin diseases, such as psoriasis, diabetic wounds, etc.^22^, ^23^ Thus, we conducted a bibliometric analysis of pertinent literature concerning the microbial immune microenvironment in melanoma during the last decade. This analysis aims to consolidate prior research, identify current trends, and offer insights to guide both scientific research and clinical applications.

The article "A bibliometric analysis of global research on microbial immune microenvironment in melanoma from 2012 to 2022" was retracted in 2025. Reasons: unreliable results or conclusions; concerns about the data.

A bibliometric analysis was performed on global publications and citations encompassing the microbial immune microenvironment in melanoma from 2012 to 2022. The scrutiny revealed an overall upward trajectory in both publication and citation numbers over the past decade, notably accelerating after 2020, with a minor dip in 2022 (Figure 2A). This signifies the recent emergence of the microbial immune microenvironment in melanoma as a prominent research subject. Leading the publication, citation, and H‐index rankings were China and the United States (Figure 2B). Furthermore, examining the cooperation network and hotspot maps of various nations, China and the United States stood out as central nodes within the collaboration network, closely engaged with countries such as Germany, France, the United Kingdom, and Finland (Figure 3A). Notably, while the United States (*n* = 80, *n* = 10 595) and China (*n* = 62, *n* = 3830) secured the top positions in terms of publication and citation volumes, Switzerland (*R* = 655) and France (*R* = 334.6) have the most outstanding average citation rates (Table 1), followed by the United States (*R* = 132.4) and China (*R* = 61.7). This indicates that although Switzerland and France have fewer publications, their research output has been recognized by scholars worldwide. Consequently, while China and the United States excel in publication quantity, Switzerland and France prioritize the quality of their articles, rendering them valuable reference points for scholars in China and the United States to draw insights from.

Regarding publication institutions (Table 2), HARVARD UNIVERSITY (*n* = 12), the UNIVERSITY OF CALIFORNIA SYSTEM (*n* = 10), and the UNIVERSITY OF TEXAS SYSTEM (*n* = 10) emerged as the leading three in publication quantity. Correspondingly, the top three in citation counts were INSTITUT NATIONAL DE LA SANTE ET DE LA RECHERCHE MEDICALE INSERM (*n* = 2820), UNIVERSITY OF TEXAS SYSTEM (*n* = 2519), and HARVARD UNIVERSITY (*n* = 1959) (Figure 3B). Among these, the INSTITUT NATIONAL DE LA SANTE ET DE LA RECHERCHE MEDICALE INSERM from France stood out not only for the highest citation count but also for the highest average citation count. The collaboration network and heatmap between institutions showed that the HARVARD MEDICAL SCHOOL was located in the center of collaborations between institutions (Figure 3C, D). It is noteworthy that within the top ten institutions with the highest publication rates, seven were based in the United States, two were in China, and one was located in France. This highlights the preeminent position of the United States in this particular domain.

The article "A bibliometric analysis of global research on microbial immune microenvironment in melanoma from 2012 to 2022" was retracted in 2025. Reasons: unreliable results or conclusions; concerns about the data.

In the distribution of authors, Zhuhao Gu from China stands out with the highest publication count (*n* = 5), whereas Jennifer A Wargo from the United States holds the record for the most citations (*n* = 943) and the highest average citation rate (*R* = 235.8) (Table 3). Gu and Steinmetz feature prominently in the central nodes of the author collaboration network across various countries (Figure 4A). In their study, Wargo et al. ^24^ conducted preclinical investigations examining fecal microbiota, dietary habits, and the use of commercial probiotic supplements in melanoma patients. The results indicated a significant association between higher dietary fiber intake and improved progression‐free survival among 128 ICB (Gut bacteria modulate the response to immune checkpoint blockade) patients. Notably, the most pronounced benefit was observed in patients with adequate dietary fiber intake who did not use probiotics, with the same outcomes validated in animal experiments. Likewise, Jennifer et al. ^25^ highlighted the pivotal role of gut microbiota in regulating overall immunity and immunotherapy for melanoma. The use of FMT (fecal microbiota transplant) has been extended to the group of melanoma patients receiving immunotherapy, which can enhance the effect of immunotherapy by enhancing the response and/or improving toxicity.

Regarding publication venues (Table 4), ADVANCED MATERIALS, CANCERS, and NATURE COMMUNICATIONS emerged as the preeminent journals, each featuring five publications in this field. Analyzing the collaboration network graph and the heat map of various journals, it becomes apparent that ADVANCED MATERIALS, FRONTIERS IN IMMUNOLOGY, and CANCERS hold central positions within the international cooperation network (Figure 4C, D). Notably, SCIENCE exhibits a significantly higher citation count (*n* = 5009) and an impressive average citation rate (*R* = 1252.2) compared to its counterparts (Figure 4B). All of the top 10 journals with the highest publications belong to JCR Q1.

Utilizing burst analysis on references (Figure 5B), a recent publication by Sivan A. stood out with the highest burst strength (3.08). As elucidated by Sivan A,^12^ Bifidobacterium holds the potential to enhance anti‐tumor immune responses by interacting with the intestinal immune system, consequently boosting the effectiveness of PD‐L1 inhibitors and successfully suppressing melanoma growth. This suggests a strategy for using probiotics to enhance the effectiveness of immunotherapy. In a similar vein, Dong and colleagues^10^ demonstrated that manipulating the composition and functionality of the gut microbiota can bolster the effectiveness of drugs used in tumor treatment, leading to increased tumor necrosis and apoptosis, effectively inhibiting melanoma growth. The inter‐referenced network diagram is shown in Figure 5A. In addition, based on the co‐citation clustering analysis of the references, a total of 14 clusters were identified, including rational combination, advanced melanoma resistance mechanism, regulating intestinal microbiota, bacteria‐based cancer therapy, gut microbiota, regulatory antitumor, PDL‐1 pathway, and cancer cell, among others (Figure 5C). According to the timeline co‐citation clustering analysis, researchers have been focusing more on the areas of gut microbiota, rational combination, and advanced melanoma resistance mechanism in recent years (Figure 5D).

The article "A bibliometric analysis of global research on microbial immune microenvironment in melanoma from 2012 to 2022" was retracted in 2025. Reasons: unreliable results or conclusions; concerns about the data.

Lastly, in the analysis of keyword co‐occurrence networks, “immunotherapy” and “cancer” are positioned centrally (Figure 6A), whereas “melanoma” and “cancer immunotherapy” feature prominently in the co‐occurrence network of author keywords (Figure 6B). Based on this, keyword clustering analysis was performed, and a total of eight keyword clusters were identified, including cancer immunotherapy, gut microbiota, drug delivery, tumor microenvironment, anticancer therapy, and drug resistance (Figure 6C). Furthermore, according to the time‐axis analysis of the reference literature keyword clustering, researchers have paid more attention to research areas such as target, gut microbiome, ipilimumab, and biomarkers in recent years (Figure 6D). Finally, citation and co‐citation analyses were conducted. Table 5 showcases the top 10 highly cited articles. The most cited article, published in Science (IF = 63.83) in 2018, has garnered 2716 citations. The central focus of this study ^26^ highlights that ICIs targeting the PD‐1/PD‐L1 axis may display anomalies in a small subset of patients, primarily due to an aberrant composition of the gut microbiome. Remarkably, administering FMT to tumor‐bearing mice significantly enhances the drug's anti‐tumor efficacy. Table 6, on the other hand, outlines the top 10 co‐cited articles, with the most co‐cited piece, published in Science (IF = 63.83) in 2018, having amassed 25 co‐citations. This particular study^19^ scrutinized the oral and gut microbiota of melanoma patients undergoing PD‐1 therapy and found that patients with a healthy gut microbiota had significantly better anti‐tumor immunity than the control group, indicating the important role of immune therapy and patient's gut microbiota characteristics in the treatment of melanoma. In addition to this, the promotion of angiogenesis by stem cell extracellular vesicles has been implicated in tumorigenesis.^27^

The article "A bibliometric analysis of global research on microbial immune microenvironment in melanoma from 2012 to 2022" was retracted in 2025. Reasons: unreliable results or conclusions; concerns about the data.

All in all, this investigation utilized the WoSCC database to identify pertinent literature concerning the microbial immune microenvironment in melanoma over the preceding decade, undertaking a thorough analysis of prevailing trends. Nonetheless, this study is not without its constraints. For instance, our scope was confined to English‐language publications, potentially overlooking numerous non‐English works. Therefore, fostering collaborations across multiple centers involving researchers from diverse nations could facilitate broader and more profound investigations. The outcomes of our study offer valuable guidance for advancing scientific research in this domain and for informing clinical approaches.

## 5 CONCLUSION

This study conducted a thorough quantitative and qualitative evaluation of publications concerning the microbial immune microenvironment in melanoma spanning 2012–2022. The quantity of publications relevant to the microbial immune microenvironment in melanoma has notably surged over the last decade, emphasizing the microbiome's role in tumor immunity as a pivotal research area for the future.

## CONFLICT OF INTEREST STATEMENT

The authors declare that the research was conducted in the absence of any commercial or financial relationships that could be construed as a potential conflict of interest.

## ETHICS STATEMENT

The authors declare human ethics approval was not needed for this study.

## Data Availability

The original contributions presented in the study are included in the article. Further inquiries can be directed to the corresponding authors.
